# Effect of Hypertonic Saline Solution Combined with Furosemide on Acute Heart Failure: A Meta-Analysis

**DOI:** 10.1155/2022/5728967

**Published:** 2022-09-21

**Authors:** Zuoqing Li, ZuanJin Wang, Nanchao Liu, Haili Li

**Affiliations:** ^1^ICU, Chengmai County People's Hospital, Chengmai 571900, China; ^2^Department of Emergency, 928th Hospital of PLA Joint Logistics Support Force, Haikou 570216, China; ^3^Department of Geriatrics, Hainan Western Central Hospital, Danzhou, 571700, China

## Abstract

**Background:**

The efficacy of hypertonic saline solution (HSS) combined with furosemide in treating acute heart failure is controversial. This meta-analysis explores the efficacy of HSS combined with furosemide for the treatment of acute heart failure.

**Methods:**

Literature were searched from databases, including PubMed, Web of Knowledge, Embase, Central, CMKI, Wanfang, and VIP. The inclusion criteria were as follows: (1) subjects: patients with acute heart failure; (2) the experimental group and the control group were properly set up; (3) intervention measures: patients in the experimental group were treated with HSS + furosemide, and patients in the control group were treated with furosemide; (4) the outcomes included at least one of the following indicators: readmission rate, mortality, 24 h urine volume, weight loss, and serum creatinine; and (5) randomized controlled trial (RCT). The method recommended by Cochrane Collaboration Network was used to evaluate the risk bias. The heterogeneity among the studies was evaluated through the chi-square test, and the publication bias was assessed by the Egger test. The results were described using risk ratio (RR), mean difference (MD), and 95% confidence interval (CI).

**Results:**

The readmission rate in the HSS + furosemide group was lower than that in the furosemide group (RR = 0.53, 95% CI [0.46, 0.60], *P* < 0.00001), with no heterogeneity among the literature (*P* = 0.21, *I*^2^ = 29%). Patients in the HSS + furosemide group had a lower mortality rate than that in the furosemide group (RR = 0.55, 95% CI [0.46, 0.65], *P* < 0.00001). The chi-square test result indicated no heterogeneity among the literature (*P* = 0.25, *I*^2^ = 23%). Furthermore, the 24 h urine volume of patients in the HSS + furosemide group was higher than that in the furosemide group (MD = 497.29, 95% CI [457.61, 536.96], *P* < 0.00001). There was no heterogeneity among the literature (*P* = 0.58, *I*^2^ = 0%). In contrast, patients in the HSS + furosemide group demonstrated a lower serum creatinine level than those in the furosemide group (MD = −0.45, 95% CI [-0.51, -0.39], *P* < 0.00001). However, heterogeneity was observed among the literature (*P* < 0.00001, *I*^2^ = 81%). The weight loss in the HSS + furosemide group was higher than that in the furosemide group (MD = 1.83, 95% CI [1.51, 2.15], *P* < 0.00001). There was no heterogeneity among the literature (*P* = 0.42, *I*^2^ = 2%). Egger test showed no publication bias among the literature (*P* > 0.05).

**Conclusion:**

Despite the heterogeneity and bias in our study, the combination of HSS with furosemide is promising in patients with acute heart failure. However, further research is still needed to confirm.

## 1. Introduction

The incidence rate and mortality of acute heart failure have steadily increased due to aging populations [1, 2]. The general purpose of treatment is to improve the symptoms of acute heart failure, stabilize hemodynamics, maintain important organ functions, avoid the recurrence of acute heart failure, and improve the long-term prognosis [3–5]. Therefore, a customized individual treatment plan should be formulated according to the inducement, severity, and classification of basic cardiovascular disease and acute heart failure [6–8].

The main measures for treating acute heart failure include cardiotonic, diuretic, and vasodilation [9, 10]. The use of diuretics can reduce edema symptoms and preload. However, about 1/3 of patients may have diuretic resistance during treatment [9, 10]. Hence, the diuretic effect of diuretics is weakened or disappeared before reaching the treatment goal of reducing edema [11–14]. Diuretic resistance is independently associated with total mortality, sudden death, and death from pump failure [15, 16]. It is necessary to increase diuretics or use multiple diuretics in combination to cope with diuretic resistance. Excessive use of diuretics may accelerate the deterioration of renal function [15–18].

Some studies [15, 18, 19] have demonstrated that furosemide combined with hypertonic saline solution (HSS) could protect patients' renal function, thus increasing diuretic effect and benefiting patients. However, the efficacy of HSS combined with furosemide in treating acute heart failure is controversial. Some studies [20] pointed out that the curative effects of combined use of HSS and simple use of furosemide on patients were similar since researchers observed no significant difference in serum creatinine level, body weight, and urine output between the two treatment regimens. Therefore, this study aims to conduct a meta-analysis to explore the efficacy of HSS combined with furosemide in treating acute heart failure.

## 2. Methods

### 2.1. Literature Search

The literature search was conducted in the following databases, including PubMed, Web of Knowledge, Embase, Central, CMKI, Wanfang, and VIP. The starting and ending time of the literature search was from the establishment of the database to June 16, 2022. There was no restriction on the language of documents.

### 2.2. Literature Screening

The inclusion criteria were as follows: (1) subjects: patients with acute heart failure; (2) the experimental group and the control group were set up; (3) intervention measures: patients in the experimental group were treated with HSS + furosemide, and patients in the control group were treated with furosemide; and (4) the outcomes included at least one of the following indicators: readmission rate, mortality, 24 h urine volume, weight loss, and serum creatinine, the readmission rate was the primary endpoint, and the remaining indicators were secondary endpoints; and (5) randomized controlled trial (RCT).

The exclusion criteria were as follows: (1) animal experiment, (2) repeated publications, (3) case reports or expert comments, (4) unable to get a full text, and (5) key data are missing and could not be supplemented by the contact author.

### 2.3. Literature Evaluation and Data Extraction

Two researchers independently reviewed and evaluated the title. They abstracted each RCT according to the identified retrieval strategy to select the literature that met the inclusion criteria. The bias risk assessment of the selected RCTs adopted the method recommended by the Cochrane Collaborative Network, namely, ① whether the random allocation method was appropriate, ② whether the blind method was adopted, ③ whether the allocation was concealled, ④ whether the baseline was comparable, and ⑤ whether to describe withdrawal and loss of follow-up. Based on the above criteria, the included studies were divided into three levels: ① low bias: all quality evaluation criteria were fully met, ② unclear: any one or more quality evaluation criteria were only partially satisfied, and ③ high bias: any one or more of the quality evaluations were completely unsatisfactory. The extracted data mainly included the first author, year of publication, number of cases, country, intervention measures, baseline characteristics, and outcome indicators. After completing the above work, two researchers crosschecked and resolved their differences through discussion.

### 2.4. Statistical Analysis

RevMan5.2 software was used to consolidate and analyze the data. The chi-square test was used to determine whether there was heterogeneity among the studies. The judgment criteria were as follows: if *P* ≥ 0.1 and *I*^2^ ≤ 50%, it was considered that there was no heterogeneity between the literature, and the fixed effect model was used for analysis. The larger the sample size, the larger the variance of the effect size, and the larger the corresponding weight distribution. If *P* < 0.1 and *I*^2^ > 50%, it was considered that there was heterogeneity between literature, and the random effect model was selected. Subgroup analysis was used to analyze the sources of heterogeneity. The publication bias was evaluated by the Egger test. Count data and measurement data were expressed in risk ratio (RR) and mean difference (MD), respectively. There is a 95% confidence interval (CI) of the calculated results. Two-way *P* < 0.05 indicates statistically significant.

## 3. Results

A total of 834 literature were obtained through database retrieval, 824 literature were excluded, and 10 studies were finally included. The flow chart of literature screening is shown in Figure 1. 10 articles included 2781 patients with acute heart failure. Among them, 1388 patients were in the HSS + furosemide group, and 1393 patients were in the furosemide group. The basic characteristics of the literature and the bias risk assessment are shown in Table 1.

### 3.1. Impact of HSS on Readmission Rate

7 articles compared the readmission rates of patients in the HSS + furosemide group and the furosemide group. The heterogeneity test results (*P* = 0.21, *I*^2^ = 29%) indicated no heterogeneity among the literature, and the fixed effect model was used. The readmission rate in the HSS + furosemide group was lower than that in the furosemide group (RR = 0.53, 95% CI [0.46, 0.60], *P* < 0.00001), as shown in Figure 2.

### 3.2. Impact of HSS on Mortality

7 articles compared the mortality of patients in the HSS + furosemide group and the furosemide group. The heterogeneity test results (*P* = 0.25, *I*^2^ = 23%) indicated no heterogeneity among the literature, and the fixed effect model was used. The mortality of the HSS + furosemide group was lower than that of the furosemide group (RR = 0.55, 95% CI [0.46, 0.65], *P* < 0.00001), as shown in Figure 3.

### 3.3. Effect of HSS on 24 h Urine Volume

The 24 h urine volume of patients in the HSS + furosemide group and the furosemide group was compared in 10 literature. The heterogeneity test results (*P* = 0.58, *I*^2^ = 0%) indicated no heterogeneity among the literature, and the fixed effect model was used. The 24 h urine volume in the HSS + furosemide group was higher than that in the furosemide group (MD = 497.29, 95% CI [457.61, 536.96], *P* < 0.00001), as shown in Figure 4.

### 3.4. Effect of HSS on Serum Creatinine

The serum creatinine levels of the HSS + furosemide group and the furosemide group were compared in 10 literature. The heterogeneity test results (*P* < 0.00001, *I*^2^ = 81%) indicated heterogeneity among the literature, and the random effect model was used. Serum creatinine in the HSS + furosemide group was lower than that in the furosemide group (MD = −0.45, 95% CI [-0.51, -0.39], *P* < 0.00001), as shown in Figure 5.

### 3.5. Effect of HSS on Weight Loss

The weight loss of the HSS + furosemide group and the furosemide group was compared in 10 literature. The heterogeneity test results (*P* = 0.42, *I*^2^ = 2%) indicated no heterogeneity among the literature, and the fixed effect model was used. The weight loss in the HSS + furosemide group was higher than that in the furosemide group (MD = 1.83, 95% CI [1.51, 2.15], *P* < 0.00001), as shown in Figure 6.

### 3.6. Publication Bias Assessment

Egger test showed no publication bias in readmission rate, mortality, 24 h urine volume, serum creatinine, and weight loss (*P* > 0.05).

## 4. Discussion

Our meta-analysis showed that HSS combined with furosemide could increase 24 h urine volume and reduce body weight and serum creatinine level in patients with acute heart failure. Patients treated with HSS combined with furosemide had a lower readmission rate and mortality than patients treated with furosemide alone.

Wan et al. [28] showed that HSS combined with furosemide could reduce the micturition volume and shorten the hospitalization time of patients with moderate and severe heart failure. Patients were followed up for 36 months and found that the readmission rate and mortality in the HSS + furosemide group were lower than those in the furosemide group. In addition, the treatment cost of the HSS + furosemide group was lower than that of the furosemide group. Licata et al. [19] showed that both HSS + furosemide and furosemide could more robustly increase the urine output of patients as well as the effect of HSSs combined with furosemide. Furthermore, HSS combined with furosemide could increase the serum sodium level, but furosemide had the opposite effect. While furosemide could increase the serum creatinine level, this phenomenon was not observed in the HSS + furosemide group. Both treatments increased serum uric acid levels. Their study [19] followed the patients for 31 months. They found that the readmission rate of patients treated with furosemide alone was higher, and the condition at readmission was worse than that at first admission. The mortality of patients treated with HSS + furosemide was lower than that of patients treated with furosemide. The literature published by Paterna et al. [27] in 2000 confirmed the feasibility of the clinical application of HSS + furosemide. In that study, HSS + furosemide could benefit patients in hemodynamics. The hospitalization time of the HSS + furosemide group was shorter than that of the furosemide group. The weight loss of the HSS + furosemide group was more significant. In addition, HSS could protect the renal function of patients with heart failure and reduce the grade of heart failure. This effect could be sustained for a long time. In the literature published in 2005, Paterna et al. [25] pointed out that the daily urine output and sodium output of patients in the HSS combined treatment group increased compared to patients treated with furosemide alone. Both treatment regimens reduced the level of BNP in patients. However, the BNP level decreased faster and more significantly in the HSS + furosemide group. Therefore, HSS combined therapy has shown advantages in shortening hospitalization time and reducing the readmission rate. Paterna et al. [26] also pointed out in the literature published in 2011 that the use of HSS could benefit patients with refractory heart failure for a long time. Compared with furosemide, HSS + furosemide could reduce the hospitalization time of patients. Paterna et al. [26] followed up the patients for 57 months. During the follow-up, they found that the readmission rate and mortality of patients in the HSS + furosemide group were lower than those in the furosemide group. Serum creatinine and urea nitrogen in the furosemide group were significantly higher than in the HSS + furosemide group. Parrinello et al. [23] pointed out that HSS could reduce clinical symptoms, improve renal function, and shorten the hospital stay of patients. HSS decreased serum troponin level and pulmonary capillary wedge pressure (PCWP). The study also noted that HSS did not cause myocardial damage. HSS could improve cardiac function, especially in diastolic volume and ejection fraction. Yayla et al. [20] pointed out that the efficacy of combined use of HSS and simple use of furosemide in patients was similar. There was no significant difference in serum creatinine level, body weight, and urine output between the two treatment regimens. The combined use of HSS could shorten the hospitalization time of patients. Okuhara et al. indicated that the 24 h urine volume and creatinine clearance rate of the HSS + furosemide group were greater than those of the control group, thus improving renal function. Parrinello et al. [24] illustrated that the 24 h urine output and sodium output of the HSS + furosemide group were higher than those of the furosemide group. Therefore, HSS combined with furosemide could significantly improve the renal function of patients. Both treatments can reduce PCWP, but HSS combined with furosemide is more effective. The study also indicated that BNP was positively correlated with PCWP. Issa et al. [21] studied and compared the levels of biomarkers of renal function in the HSS + furosemide group and furosemide group. They suggested that HSS + furosemide could significantly improve patients' renal function.

This study has some limitations. First, there was a risk of bias in the literature included in the analysis, which might affect the results. And there were differences in research objects and intervention measures in various literature, which might be the source of heterogeneity. Secondly, the outcome indicators included in our analysis were limited, and we could not comprehensively evaluate the efficacy of HSS combined with furosemide in patients with acute heart failure. Third, the results obtained by subgroup analysis according to age, gender, and severity of heart failure are more clinically instructive. However, we were limited by literature information and were unable to perform such subgroup analyses. Fourth, this study failed to retrieve relevant studies in recent years, and the literature included in the analysis was outdated, which may have a certain impact on the results.

In conclusion, despite the heterogeneity and bias in our study, the combination of HSS with furosemide is promising in patients with acute heart failure. However, further research is still needed to confirm.

## Figures and Tables

**Figure 1:** Document screening flow chart. RCT: randomized controlled trial.

**Figure 2:** Comparison of readmission rate between the HSS + furosemide group and the furosemide group. HSS: hypertonic saline solution.

**Figure 3:** Comparison of mortality between the HSS + furosemide group and the furosemide group. HSS: hypertonic saline solution.

**Figure 4:** Comparison of 24 h urine volume between the HSS + furosemide group and the furosemide group. HSS: hypertonic saline solution.

**Figure 5:** Comparison of serum creatinine levels between the HSS + furosemide group and the furosemide group. HSS: hypertonic saline solution.

**Figure 6:** Comparison of weight loss between the HSS + furosemide group and the furosemide group. HSS: hypertonic saline solution.

**Table 1:** Basic characteristics of literature and risk assessment of bias.

Author	Year	No. of patients		Outcomes	Risk of basis
		HSS+ furosemide	Furosemide		
Issa et al. [21]	2013	20	12	Urine output, length of stay, readmission rate, hospitalization cost, mortality, readmission time	Uncertain
Licata et al. [19]	2003	53	54	Urine output, serum creatinine, readmission rate, mortality, body weight	Uncertain
Okuhara et al. [22]	2014	22	22	Urine output, brain natriuretic peptide, natriuretic capacity, length of hospital stay, readmission rate, mortality	Low
Parrinello et al. [23]	2012	66	67	Length of hospital stay, readmission, and mortality	Uncertain
Parrinello et al. [24]	2011	122	126	Urine volume, serum creatinine, readmission rate, length of hospital stay, natriuretic capacity, body weight, mortality	Uncertain
Paterna et al. [25]	2005	30	30	Brain natriuretic peptide, body weight, urine volume, serum creatinine	Uncertain
Paterna et al. [26]	2011	48	46	Serum creatinine, body weight, length of stay, readmission rate	Uncertain
Paterna et al. [27]	2000	881	890	Urine volume, serum creatinine, body weight, readmission rate, mortality	Uncertain
Wan et al. [28]	2017	132	132	Urine volume, serum creatinine, body weight, brain natriuretic peptide	Uncertain
Yayla et al. [20]	2015	14	14	Urine volume, serum creatinine, body weight	Low

Note: HSS: hypertonic saline solution.

## Data Availability

The data used and analyzed during the current study are available from the corresponding author.
